# Versatile Production of Poly(Epsilon-Caprolactone) Fibers by Electrospinning Using Benign Solvents

**DOI:** 10.3390/nano6040075

**Published:** 2016-04-15

**Authors:** Liliana Liverani, Aldo R. Boccaccini

**Affiliations:** Institute of Biomaterials, Department of Materials Science and Engineering, University of Erlangen-Nuremberg, Cauerstr. 6, 91058 Erlangen, Germany; aldo.boccaccini@fau.de

**Keywords:** electrospinning, benign solvents, nanofibers, poly(epsilon-caprolactone), macroporosity, composite, bioactive glass

## Abstract

The electrospinning technique is widely used for the fabrication of micro- and nanofibrous structures. Recent studies have focused on the use of less toxic and harmful solvents (benign solvents) for electrospinning, even if those solvents usually require an accurate and longer process of optimization. The aim of the present work is to demonstrate the versatility of the use of benign solvents, like acetic acid and formic acid, for the fabrication of microfibrous and nanofibrous electrospun poly(epsilon-caprolactone) mats. The solvent systems were also shown to be suitable for the fabrication of electrospun structures with macroporosity, as well as for the fabrication of composite electrospun mats, fabricated by the addition of bioactive glass (45S5 composition) particles in the polymeric solution.

## 1. Introduction

Electrospinning is a well-established technique widely used for the fabrication of micro- and nanofibrous mats for numerous applications, including for the biomedical field, e.g. drug delivery and tissue engineering scaffolds. The principle at the basis of the electrospinning process is the application of a high voltage at the tip of a needle containing a polymer solution, suspension, blend or melt. During the time of flight the solvent evaporates from the charged solution and the obtained fibers are collected on the grounded target. The electrospinning process and the characteristics of the obtained electrospun mats are affected by several parameters. They could be grouped in three categories: solution parameters, process parameters and environmental parameters [1,2,3].

In the tissue engineering field, the versatility of this scaffold fabrication technique is proven by the increasing number of publications during the last years, by the integrated use of electrospinning with other scaffold fabrication techniques and by the development of a high number of different electrospinning setups [1]. A huge number and variety of polymers can be processed by electrospinning, but often the use of organic toxic solvents is required. Recently, the introduction of the “Green Electrospinning” concept [4] and the awareness about the disadvantages related to the use of toxic solvents, as environmental impact, safety related issues for the lab workers and the possible presence of residuals of toxic solvents in the electrospun mats, have raised the interest in the use of less or not toxic solvents (benign solvents) for electrospinning [5,6].

Poly(epsilon-caprolactone) (PCL) is a biodegradable linear aliphatic polyester which is widely used for tissue engineering, biomedical, food and other industrial applications [7,8,9]. PCL usually exhibits a low degradation rate in aqueous solution, with non-toxic products of degradation. Even if its hydrophobicity cannot promote and allow cell adhesion, it is possible to post-treat the sample in order to modify its surface without affecting the fibrous structure, and different types of treatments are already reported in literature [10,11,12]. It is also possible to blend PCL with other polymers in order to modulate its properties [13,14,15].

Since the beginning of the spreading of the electrospinning technique, PCL, other polyesters and their blends have been processed by this method [16,17]. PCL is soluble in tetrahydrofuran, chloroform, methylene chloride, carbon tetrachloride, benzene, toluene, cyclohexanone dihydropyran and 2-nitropropane and only partially soluble in acetone, 2-butanone, ethyl acetate, acetonitrile and dimethyl fumarate [18,19]. For the electrospinning process, it is common to solve PCL using mixtures of solvents and co-solvents, like chloroform/methanol, methylene chloride/methanol, methylene chloride/N,N-dimethylformamide (DMF), methylene chloride/toluene or tetrahydrofuran/DMF [20,21,22,23]. Unfortunately most of these solvents suitable for electrospinning are toxic and harmful, for this reason, recently several research works have focused on the use of less toxic and harmful solvents for electrospinning, *i.e.* acetic acid, formic acid and acetone [5,24,25,26]. These studies have demonstrated the increased focus on less harmful solvents for electrospinning but they have also highlighted that most of these solvents are not directly suitable for electrospinning, requiring a longer and more accurate optimization of the process.

For tissue engineering applications, considering the importance of mimicking the native structure and function of the extracellular matrix (ECM), the electrospinning technique is particularly relevant for the obtainment of nanosized fibers [1]. As already reported in literature by Soliman *et al.* [20], it is possible to obtain PCL nano- and microfibers by just regulating and adjusting the polymeric solution concentration without changing solvents, however in such cases the solvent is usually a mixture of chloroform and methanol. Recently, other studies have considered the fabrication of PCL nanofibers using less harmful solvents, like formic acid. In fact, formic acid is relevant for the reduction of the fiber diameter, as already reported by Van der Schueren *et al.* [24], who showed that the increase of the amount of formic acid in the electrospinning solution leads to a decrease in the average fiber diameter.

The relevance of the presence of macroporosity in electrospun fiber mats has been highlighted by the need of pores able to allow cell infiltration inside the electrospun mats and, considering the density of the fibrous structure, often cells could only adhere on the surface without penetrating inside the mesh [2,7]. The dimension and the interconnectivity of the porosity are crucial elements for tissue engineering scaffolds and they are also related to the cell type and the target tissue [27].

The electrospinning technique has been widely used to pursue a biomimetic approach to obtain composite structures [28] in order to reproduce the composition of native tissue. In fact the suitability of the electrospinning of suspensions containing inorganic phases in the polymeric solutions has been already investigated for bone tissue engineering applications [29,30]. In particular, for this goal, the use of bioactive glass (BG) particles is relevant to promote mineralization of the constructs and also because of the BG bioactivity, and its effect on osteogenesis and angiogenesis processes [31].

In this framework, the aim of the present work has been the optimization of the electrospinning of poly(epsilon-caprolactone) (PCL) using acetic acid and a mixture of acetic acid and formic acid as solvents, demonstrating the feasibility of producing bead-free micro- and nanofibers with the use of such benign solvents. Beyond the electrospinning process optimization, the novelty of the present work resides in the evaluation of the suitability of these solvents for the fabrication of patterned mats, which allows the formation of macroporosities relevant for improving cell infiltration inside the electrospun mats. In addition, the versatility of the solvents for the fabrication of composite fibers, obtained with the addition of bioactive glass particles inside the polymeric solution, was considered in order to obtain organic-inorganic composite electrospun mats suitable for bone tissue engineering applications.

## 2. Results and Discussion

### 2.1. Influence of Solution Parameters

To evaluate the suitability for electrospinning of solutions of PCL dissolved in acetic acid, different solutions were tested and the electrospinning parameters were kept constant, , as reported in the experimental section. In particular, PCL was solved in glacial acetic acid at concentrations of 12%, 15%, 18% and 20% *w*/*v*. As already reported in the literature [25], the solution parameters affect the morphology of the obtained mats. In fact, with low polymer concentration (12% and 15% *w*/*v*), we have obtained electrospun mats full of beads, as shown in Figure 1A,B. Differences between the two samples can be observed; it was noted that increasing the amount of polymer the shape of the beads became less round and more spread (spindle-like shape). The fiber diameter was also seen to increase by increasing the amount of PCL in the solution. In the sample obtained with the 18% *w*/*v* solution (Figure 1C), it is possible to observe a reduction in the number of beads and defects in the mesh, respect to the sample obtained from the 12% and 15% solutions, also confirming the increasing trend in fiber diameter, showing a significant inhomogeneity in the distribution of the fiber average diameter, as reported in Table 1. All samples having an amount of PCL less than 20% *w*/*v* showed a non-homogeneous distribution of the fiber average diameter, as reported in Table 1 and Figure 1. The solution of 20% *w*/*v* PCL showed a homogeneous defect-free electrospun fiber mat confirming the relationship between polymer amount and fiber diameter, as shown in Figure 2.

All measured values of fiber diameters are two or three times lower with respect to similar samples reported in literature [5,25]. In fact, Ferreira and *et al.* [5] reported an average fiber diameter of 1.96 ± 0.52 μm for mats obtained from a solution of 20 wt % of PCL in acetic acid, with a flow rate of 0.4 mL/h and an applied voltage of 6 kV and Kanani *et al.* [25], starting from a solution of 20% PCL in glacial acetic acid, reported a range of average fiber diameters between 2.5 and 3 μm, with an applied voltage of 15 kV and a flow rate of 0.5 mL/h. The shape and the size of the beads in samples obtained from a solution of PCL 12% *w*/*v* are comparable to the beads size reported by Kanani *et al.* [25] for a solution of 10% PCL, even if the fiber average diameter is slightly different.

### 2.2. Influence of the Applied Voltage

Starting from the solution of 20% *w*/*v* of PCL in acetic acid, an evaluation of the influence of the electrospinning process parameters has been performed. The parameter found to be the most relevant was the applied voltage: keeping constant all the other process parameters, applied voltages of 10, 15 and 20 kV were applied and the obtained mats are reported in Figure 3. It is possible to notice that beads-free electrospun mats have been obtained for all conditions. For the lowest value of the applied voltage, the fiber diameter is not homogeneous and it is possible to see discontinuities inside the mats (Figure 3A). On the other hand, the fibers obtained using the highest value of applied voltage started to blend and the yield of the electrospinning process itself was reduced in comparison to the other two samples.

### 2.3. Optimization of Solvent Mixture for Obtaining Nanofibers

Fabricating nanofibrous structures is relevant for tissue engineering applications due to their structural similarity with the native ECM and the expected enhancement in cell spreading, even if thick layer of nanofibers cannot allow cell infiltration and migration within the mats [32].

The use of formic acid for electrospinning PCL has been already associated in the literature to a reduction in average fiber diameter of the obtained mats [24]. In the present work the addition of formic acid to the PCL solution was performed in order to produce homogeneous nanofibrous mats, since with the use of acetic acid alone it was not possible to achieve an homogeneous distribution of fiber diameters in the nanoscale, as shown in Figure 4. Compared to the literature [24], by comparing a similar polymer concentration of the starting solution with greater amounts of acetic acid and with different electrospinning parameters, in the present work, fibers exhibiting two times lower average fiber diameters were obtained. In fact, PCL nanofiber mats were obtained by keeping constant the value of the PCL concentration at 15% *w*/*v* with the addition of formic acid (in ratio 1:1 to acetic acid) and optimizing the electrospinning parameters. The average fibers diameter was 0.20 ± 0.04 μm, while the similar sample without formic acid exhibited an average fiber diameter of 0.3 ± 0.2 μm. SEM micrographs of both samples are shown in Figure 4.

### 2.4. Macroporosities in Electrospun Fiber Mats

As reported by Ferreira *et al.* [5], the porosity usually obtained in electrospun mats intended as tissue engineering scaffolds is not sufficient to reach the goal of an effective cell infiltration inside the mats. The need for macropores in electrospun mats has been widely reported and explained in literature [7,27,33]. For this reason, in this study about the versatility of production of PCL electrospun fibers using benign solvents, the fabrication of macropores in the electrospun mats was investigated.

PCL microfibers, obtained with the PCL solution of 20% *w*/*v* in acetic acid (sample PCL20_AA_15), were obtained using the same electrospinning parameters, and applying a patterned target, as shown in Figure 5. The fibers morphology was not affected by the different targets used and, even if few fibers are visible inside the pores, well-defined macropores of square shape and average size of 0.47 ± 0.08 mm were obtained.

The duration of the electrospinning process has a crucial role and it affects the opening of the macroporosities; in fact, by increasing the time of the process, the electrospun mats progressively covered the patterned collector closing the macroporosities, as already reported [34].

For the nanofibers (sample PCL15_AAFA), the same patterned collector used for microfibers was employed, but it was noticed that a reduced time of electrospinning was necessary for formation of the patterned mesh, shown in Figure 6A. This reduced time implies also a reduced thickness of the mats, posing issues in the mats handling. In addition, another patterned collector with a wider net was used with the nanofibers in order to obtain better results in terms of mats thickness. However, with the wider nets, it was not possible to achieve open macropores and the electrospun mats covered completely the patterned target, maintaining the morphology of the pattern, as shown in Figure 6B.

### 2.5. Composite Electrospun Fibers

The addition of BG particles to the PCL solution before electrospinning was investigated to evaluate the suitability of the benign solvents for electrospinning, as well as to demonstrate the versatility of the approach for the fabrication of composite fibrous mats.

The average fiber diameter has been reported to increase with the addition of nanoparticles [35,36,37], since the viscosity of the solution usually increases by the presence of the particles. In the present work, an increase in the solution viscosity was also observed and the electrospinning parameters (like flow rate and needle diameter) were adapted and optimized on the new solution containing BG particles, as reported in the experimental section. The obtained results are presented in Figure 7A–C; SEM micrographs show a decrease in fiber average diameter, that is 0.5 ± 0.2 μm, and an increase in the inhomogeneity of the fiber diameter distribution, compared to the neat PCL mats (average fiber diameter 1.0 ± 0.1 μm). BG particles are visible inside the electrospun mats, in particular in Figure 7B,C, it is possible to notice that the particles size is also maintained (about 2 μm). By considering energy dispersive X-ray (EDX) analysis results, reported in Figure 8, in the d0 sample, it is also possible to identify BG particles because of their Si content.

After the first day of immersion in simulated body fluid (SBF) solution (Figure 7D–F), it was possible to notice that the PCL-BG composite fibers are already covered by precipitated mineral phase. It is possible to observe that not only the BG particles, but also all of the fibers started to be homogeneously covered by the deposits, however the samples fibrillar structure was preserved. In the following time points, it was apparent that the fibers and also the BG particles were completely covered by precipitates (Figure 7G–I). In the last time point, the electrospun mats resulted completely covered and some artifacts were observed (Figure 7L–N). A progressive and complete covering of the electrospun mats is observed, while the mats maintain their fibrous structure, however with increasing the time of immersion in SBF solution it is also evident that it is not easy to wash and remove some deposits (artifacts) embedded inside the fibrous mats. The neat PCL mats were also immersed in SBF, as control. As shown in Figure 7, it was confirmed that no deposition of a mineral phase on the neat PCL sample occurred. The combination of SEM observations and Fourier transform infrared spectroscopy (FTIR) analysis is necessary to clarify the nature of such precipitates on the samples. EDX analysis was also performed to characterize the nature of the precipitates on the fibers and results are reported in Figure 8, in which it is possible to notice the progressive increase in the amount of calcium and phosphorus with increasing time of immersion in SBF solution. In particular, when the data are normalized with respect to the amount of Carbon (main component due to the polymer), an increase in the presence of Ca and P at the different time points of immersion in SBF solution becomes apparent. The ratio Ca/P is constant at the different time points (d1, d4 and d7) and the Ca/P ratio value lies between a minimum of 1.8 and a maximum of 2.0.

### 2.6. ATR-FTIR Analysis

ATR-FTIR analysis was used for the assessment of the influence of the solvent on the obtained electrospun mats chemical composition, for the evaluation of the presence of BG inside the sample and for the confirmation of sample *in vitro* bioactivity. In Figure 9 and Figure 10, the FTIR spectra of neat PCL, and PCL-BG before (PCL-BG d0) and after immersion in SBF solution (PCL-BG d1 and PCL-BG d4) are reported. No differences between the IR spectra of microfibrous and nanofibrous neat PCL samples have been recorded, and for this reason just one spectrum was included in Figure 9 and Figure 10. In addition, the PCL-BG sample immersed in SBF for seven days showed the same bands reported in the spectrum of the sample immersed for four days (PCL-BG d4).

All spectra exhibit the main PCL bands, as shown in Figure 9, including the two peaks centered around 2943 cm^−1^ and 2866 cm^−1^ due to asymmetric and symmetric CH_2_ stretching, respectively, the peak at 1722 cm^−1^ ascribable to carbonyl stretching, the peak at 1294 cm^−1^ due to C–O and C–C stretching and the peaks centered around 1240 and 1165 cm^−1^, due to asymmetric and symmetric C–O–C stretching, respectively [38,39,40].

The spectrum of the sample with BG particles (sample PCL-BG d0, before immersion in SBF) is also characterized by the main PCL bands. A band due to Si-O-Si stretching vibration centered around 1190 cm^−1^ is detectable in PCL-BGd0 spectrum as a shoulder, since it is overlapped with the PCL bands, and it is visible in the subtraction spectrum (PCL-BGd0–PCL, not shown).

The sample bioactivity (given by the ability of the material to induce the formation of hydroxyapatite on its surface [41]) has been tested by immersion in SBF solution. Already after one day of immersion (PCL-BG d1, spectrum reported in Figure 10) it is possible to notice a reduction in the intensity of the peaks centered around 1165 and 1045 cm^−1^. Moreover, new peaks are observed centered around 1027 cm^−1^, ascribable to PO_4_^3−^ asymmetric stretching vibration, according to [42]. In addition, the new peaks at 560 and 600 cm^−1^, are due to P–O bending vibration in crystalline phosphate, like apatite [43].

These results support the statement that the precipitates shown in the SEM micrographs in Figure 7 are associated with hydroxyapatite deposition, demonstrating that BG particles bioactivity is preserved after electrospinning, independently of the solvent used. The preservation of bioactivity after addition of BG particles in electrospinning polymeric solutions has been already reported in literature [36,44]. Even if Gönen *et al.* [35] reported that for their electrospun mats of gelatin/PCL with particles of strontium and copper doped bioactive glasses, the bioactivity was not shown by all their composite samples, it is likely that the bioactivity effect strongly depends on the amount of particles inside the starting polymer solution.

### 2.7. Mechanical Properties

Samples mechanical properties were evaluated in order to investigate a possible correlation with the fiber diameter; results are included in Table 2.

No significant differences in terms of Young’s modulus were detected from comparison between the electrospun microfibers (PCL20_AA_15) and the nanofibrous sample (PCL15_AAFA). According to the literature, Ferreira *et al.* [5] also reported that the average fiber diameter did not affect mats mechanical properties, at least in the range of 1.4–3.4 μm, and their evaluation was supported by reporting the values of Young’s modulus and showing similar stress–strain curves for all investigated samples [5]. This result is particularly relevant because, with respect to the literature [5], a wider difference between the investigated fiber size diameter (nanosized *vs.* microsized) and the possible influence on the mats mechanical properties has been evaluated.

The addition of BG particles implies a reduction in the value of Young’s modulus but it does not affect other parameters. The effect of the addition of BG particles on mechanical properties must be coupled with the reduction in the average fiber diameter, with the increase in the inhomogeneity in the distribution of the average fiber diameter and with the presence of roughness on the surface of the electrospun mats, as shown in Figure 11. In addition, lack of strong adhesion between BG particles and PCL at interfaces could have led to the reduction of Young’s modulus and ultimate tensile strength (UTS), as reported in the literature for similar composites [45].

## 3. Experimental Section

### 3.1. Synthesis

Electrospun mats were obtained from PCL (80 kDa, Sigma Aldrich, Munich, Germany) solutions. Acetic acid (AA, VWR, Darmstadt, Germany) and formic acid (FA, VWR, Darmstadt, Germany) were used as solvents.

The details of each solution (solvent and polymer concentration) are reported in Table 3. The solutions of PCL in acetic acid were stirred overnight and then were put in an ultra-sound bath for 1 hour. For the fabrication of the composite electrospun mats, commercially available BG particles (Schott Vitryxx®, size 2 μm, Schott AG, Mainz, Germany) were homogeneously dispersed (30 wt % respect to PCL) in the polymer solution and stirred for 10 minutes. The PCL solution used for PCL-BG samples was the solution containing 20% *w*/*v* of PCL in acetic acid.

### 3.2. Electrospinning Process

The optimization of the electrospinning parameters was performed and different solution concentrations and solvents systems were evaluated, as summarized in Table 3. Electrospinning was performed using a commercially available setup (Starter Kit 40KV Web, Linari Engineering srl, Valpiana (GR), Italy). The optimized electrospinning parameters for the solution of 20% *w*/*v* of PCL were an applied voltage of 15 kV, a needle-target distance of 11 cm, while the polymeric solution was fed with a flow rate of 0.4 mL/h.

### 3.3. Characterization

Samples morphology was assessed by SEM analysis (FE-SEM-EDS (Auriga 0750, Zeiss, Jena, Germany)). Samples were sputtered with gold before SEM analysis using a Sputter Coater (Q150T, Quorum Technologies, Darmstadt, Germany). Fiber average diameters were calculated using ImageJ (NIH, Bethesda, MD, USA), after the measurement of 50 fibers from each sample.

FTIR spectra of selected samples were obtained using an FTIR spectrometer (Nicolet 6700, Thermo Scientific, Schwerte, Germany) in attenuated total reflectance mode (ATR). For the analysis, 32 spectral scans at a resolution of 4 cm^−1^ were repeated over the wavenumber range 4000–550 cm^−1^. The used window material was CsI.

The mechanical characterization of selected fibrous mats was performed by uniaxial tensile strength test, by using a universal testing machine (Zugfestigkeitsprüfmaschine Frank, K. Frank GmbH, Mannheim, Germany) at room temperature. The measurements were carried out at a crosshead speed of 10 mm/min by using a 50 N load cell. In order to handle correctly the electrospun mats, avoiding the application of any pretension on the samples before the mechanical tests, the use of a suitable paper square framework was necessary. The samples were cut in rectangular shape of 5 mm wide and 4 cm long and the internal length of the paper framework was 2 cm.

The acellular bioactivity of the electrospun composite samples containing BG was evaluated by the immersion of the samples in a simulated body fluid (SBF) solution, according to the protocol reported in ref. [41], for 1, 4 and 7 days. After the immersion, the samples were characterized by SEM, EDX and ATR-FTIR analyses. Samples of neat PCL electrospun mats were used as control. The bioactivity of the samples was related to the formation of hydroxyapatite phase on the surface of samples, upon immersion in SBF [41].

## 4. Conclusions

Defect-free nanofibrous and microfibrous PCL mats were successfully fabricated by electrospinning using benign solvents. The versatility and suitability of these solvents for the electrospinning process were investigated for fabrication of electrospun mats with well-defined macroporosity, with pore size of 0.47 ± 0.08 mm, suitable for enhancing cell migration and infiltration into the electrospun mats for tissue engineering applications. The use of different targets to obtain different patterned structures was also investigated. The suitability of the solvents was also tested for the fabrication of composite electrospun structures. The obtained PCL electrospun mats containing BG particles were beads-free, preserving the BG bioactivity. Further work will be focused on the use of the obtained mats as layers of complex multilayered structures for bone and interface tissue engineering applications.

## Figures and Tables

**Figure 1:** Scanning electron microscopy (SEM) micrographs of electrospun poly(epsilon-caprolactone) (PCL) mats obtained from different PCL solutions in acetic acid (scale bar 20 μm): (**A**) 12% *w*/*v*; (**B**) 15% *w*/*v*; (**C**) 18% *w*/*v*; and (**D**) 20% *w*/*v*.

**Figure 2:** Trend of the PCL mats average fiber diameter as function of the PCL solution concentrations.

**Figure 3:** Influence of the applied voltage to the PCL solution of 20% *w*/*v* on electrospun fiber characteristics: (**A**) 10 kV; (**B**) 15 kV; and (**C**) 20 kV (scale bar 2 μm).

**Figure 4:** Representative SEM micrographs of PCL nanofibers (scale bar 2 μm): (**A**) PCL 15% *w*/*v* in acetic acid; and (**B**) PCL 15% *w*/*v* in a mixture of acetic acid and formic acid (ratio 1:1).

**Figure 5:** Light microscope image of PCL microfibers pattern (**A**). SEM micrographs of PCL microfibers pattern exhibiting large porosity at different magnifications: 100× (scale bar 100 μm) (**B**); and 200× (scale bar 100 μm) (**C**).

**Figure 6:** Light Microscope image of PCL nanofibers pattern: with the narrow pattern (magnification 4×) (**A**); and with the wide pattern (magnification 1× and in the inlet 4×, scale bar 1 mm) (**B**).

**Figure 7:** SEM micrographs of PCL and PCL-bioactive glass (BG) composite electrospun mats before immersion in simulated body fluid (SBF) solution (PCL d0 and PCL-BG d0 (**A**–**C**)) in the first row; after one day of immersion in SBF (PCL d1 and PCL-BG d1 (**D**–**F**)) in the second row; after four days of immersion in SBF (PCL d4 and PCL-BG d4 (**G**–**I**)); and after seven days of immersion in SBF (PCL d7 and PCL-BG d7 (**L**–**N**)).

**Figure 8:** Energy dispersive X-ray (EDX) analysis of PCL-BG composite electrospun mats before immersion in SBF solution (PCL-BG d0) in the first row; after one day of immersion in SBF (PCL-BG d1) in the second row; after four days of immersion in SBF (PCL-BG d4); and after seven days of immersion in SBF (PCL-BG d7).

**Figure 9:** Fourier transform infrared spectroscopy (FTIR) spectra in the range 3000–500 cm^−1^ for electrospun samples of neat PCL (PCL), PCL with BG particles before immersion in SBF solution (PCL-BG d0) and after one day (PCL-BG d1) and four days (PCL-BG d4) of immersion in SBF solution (the characteristic peaks are discussed in the text).

**Figure 10:** FTIR spectra in the range 1300–500 cm^−1^ for electrospun samples of neat PCL (PCL), PCL with BG particles before immersion in SBF solution (PCL-BG d0) and after one day (PCL-BG d1) and four days (PCL-BG d4) of immersion in SBF solution (the characteristic peaks are discussed in the text).

**Figure 11:** Digital images of electrospun fiber mats without (PCL20) and with BG particles (PCL-BG) before the mechanical testing.

**Table 1:** Summary of PCL fiber mats produced including sample name, fiber average diameter, and size of minimum and maximum fiber diameter measured on SEM micrographs (sample name: PCLsolutionconcentration_solvent_kV).

Sample	Fiber Average Diameter	Minimum Fiber Diameter	Maximum Fiber Diameter
PCL12_AA_15 *	0.12 ± 0.03 μm	0.09 μm	0.2 μm
PCL15_AA_15 *	0.18 ± 0.02 μm	0.1 μm	0.2 μm
PCL18_AA_15	1.0 ± 0.6 μm	0.3 μm	3.6 μm
PCL20_AA_15	1.0 ± 0.1 μm	0.7 μm	1.2 μm

* For these samples, the beaded fibers were not evaluated for calculating the fiber average diameter.

**Table 2:** Average fiber diameter and mechanical properties of the electrospun mats. UTS: ultimate tensile strength.

Sample Name	Average Fiber Diameter (μm)	Young’s Modulus (Mpa)	UTS (Mpa)	Tensile Strain (%)
**PCL20_AA_15**	1.0 ± 0.1	12 ± 5	1.2 ± 0.3	83 ± 10
**PCL15_AAFA**	0.20 ± 0.04	11.0 ± 0.8	6.2 ± 0.9	115 ± 2
**PCL-BG**	0.5 ± 0.2	4.2 ± 0.9	1.2 ± 0.3	90 ± 18

**Table 3:** Summary of the electrospinning parameters for the different tested solutions and indication of the related SEM micrograph showing the fiber mat microstructure.

Sample Name	Solution Concentration (% *w*/*v*)	Solvent(s)	kV	Distance Tip-Target (cm)	Needle Diameter (G)	Flow Rate (mL/h)	T (°C)	Relative Humidity (RH) (%)	SEM Micrograph
PCL12	12	AA	15	11	23	0.4	23.6	42	Figure 1A
PCL15_AA	15	AA	15	11	23	0.4	23.5	43	Figure 1B and Figure 4A
PCL15_AAFA	15	AA/FA	20	11	23	1.3	23.6	43	Figure 4B
PCL18	18	AA	15	15	23	0.4	23.5	49	Figure 1C
PCL20_10	20	AA	10	11	23	0.4	29.0	45	Figure 3A
PCL20_15	20	AA	15	11	23	0.4	28.0	48	Figure 1D and Figure 3B
PCL20_20	20	AA	20	11	23	0.4	23.5	28	Figure 3C
PCL-BG	20	AA	15	11	21	0.8	23.6	49	Figure 7A,B,C

## References

[1] Jiang T., Carbone E.J., Lo K.W.-H., Laurencin C.T. (2015). Electrospinning of polymer nanofibers for tissue regeneration. Prog. Polym. Sci..

[2] Sun B., Long Y.Z., Zhang H.D., Li M.M., Duvail J.L., Jiang X.Y., Yin H.L. (2014). Advances in three-dimensional nanofibrous macrostructures via electrospinning. Prog. Polym. Sci..

[3] Putti M., Simonet M., Solberg R., Peters G.W.M. (2015). Electrospinning poly(ε-caprolactone) under controlled environmental conditions: Influence on fiber morphology and orientation. Polymer (Guildf).

[4] Agarwal S., Greiner A. (2011). On the way to clean and safe electrospinning-green electrospinning: Emulsion and suspension electrospinning. Polym. Adv. Technol..

[5] Ferreira J.L., Gomes S., Henriques C., Borges J.P., Silva J.C. (2014). Electrospinning polycaprolactone dissolved in glacial acetic acid: Fiber production, nonwoven characterization, and *in vitro* evaluation. J. Appl. Polym. Sci..

[6] Ghosal K., Thomas S., Kalarikkal N., Gnanamanis A. (2014). Collagen coated electrospun polycaprolactone (PCL) with titanium dioxide (TiO_2_) from an environmentally benign solvent: Preliminary physico-chemical studies for skin substitute. J. Polym. Res..

[7] Dash T.K., Konkimalla V.B. (2012). Poly-ε-caprolactone based formulations for drug delivery and tissue engineering: A review. J. Control. Release.

[8] Zhang L., Xiong C., Deng X. (1995). Biodegradable polyester blends for biomedical application. J. Appl. Polym. Sci..

[9] Duncan T.V. (2011). Applications of nanotechnology in food packaging and food safety: Barrier materials, antimicrobials and sensors. J. Colloid Interface Sci..

[10] Zhu W., Castro N.J., Cheng X., Keidar M., Zhang L.G. (2015). Cold Atmospheric Plasma Modified Electrospun Scaffolds with Embedded Microspheres for Improved Cartilage Regeneration. PLoS ONE.

[11] Tiaw K.S., Goh S.W., Hong M., Wang Z., Lan B., Teoh S.H. (2005). Laser surface modification of poly(ε-caprolactone) (PCL) membrane for tissue engineering applications. Biomaterials.

[12] Marletta G., Ciapetti G., Satriano C., Perut F., Salerno M., Baldini N. (2007). Improved osteogenic differentiation of human marrow stromal cells cultured on ion-induced chemically structured poly-ε-caprolactone. Biomaterials.

[13] Cheng Z., Teoh S.H. (2004). Surface modification of ultra thin poly(epsilon-caprolactone) films using acrylic acid and collagen. Biomaterials.

[14] Da Silva G.R., Lima T.H., Oréfice R.L., Fernandes-Cunha G.M., Silva-Cunha A., Zhao M., Behar-Cohen F. (2015). *In vitro* and *in vivo* ocular biocompatibility of electrospun poly(ɛ-caprolactone) nanofibers. Eur. J. Pharm. Sci..

[15] Li X., Xie J., Yuan X., Xia Y. (2008). Coating electrospun poly(ε-caprolactone) fibers with gelatin and calcium phosphate and their use as biomimetic scaffolds for bone tissue engineering. Langmuir.

[16] Huang Z.M., Zhang Y.Z., Kotaki M., Ramakrishna S. (2003). A review on polymer nanofibers by electrospinning and their applications in nanocomposites. Compos. Sci. Technol..

[17] Yoshimoto H., Shin Y.M., Terai H., Vacanti J.P. (2003). A biodegradable nanofiber scaffold by electrospinning and its potential for bone tissue engineering. Biomaterials.

[18] Suggs L.J., Moore S.A., Mikos A.G., Mark J.E. (2007). Physical Properties of Polymers Handbook. Physical Properties of Polymers Handbook.

[19] Pitt C.G., Chasin M., Langer R. (1990). Poly-ε-Caprolactone and Its Copolymers. Biodegradable Polymers As Drug Delivery Systems.

[20] Soliman S., Sant S., Nichol J.W., Khabiry M., Traversa E., Khademhosseini A. (2011). Controlling the porosity of fibrous scaffolds by modulating the fiber diameter and packing density. J. Biomed. Mater. Res. Part A.

[21] Lee K.H., Kim H.Y., Khil M.S., Ra Y.M., Lee D.R. (2003). Characterization of nano-structured poly(ε-caprolactone) nonwoven mats via electrospinning. Polymer (Guildf).

[22] Li W.-J., Danielson K.G., Alexander P.G., Tuan R.S. (2003). Biological response of chondrocytes cultured in three-dimensional nanofibrous poly(epsilon-caprolactone) scaffolds. J. Biomed. Mater. Res. A.

[23] Prabhakaran M.P., Venugopal J.R., Chyan T.T., Hai L.B., Chan C.K., Lim A.Y., Ramakrishna S. (2008). Electrospun biocomposite nanofibrous scaffolds for neural tissue engineering. Tissue Eng. Part A.

[24] Van Der Schueren L., De Schoenmaker B., Kalaoglu Ö.I., De Clerck K. (2011). An alternative solvent system for the steady state electrospinning of polycaprolactone. Eur. Polym. J..

[25] Kanani A.G., Bahrami S.H. (2011). Effect of Changing Solvents on Poly(ε-Caprolactone) Nanofibrous Webs Morphology. J. Nanomater..

[26] Katsogiannis K.A.G., Vladisavljević G.T., Georgiadou S. (2015). Porous electrospun polycaprolactone (PCL) fibres by phase separation. Eur. Polym. J..

[27] Oh S.H., Park I.K., Kim J.M., Lee J.H. (2007). *In vitro* and *in vivo* characteristics of PCL scaffolds with pore size gradient fabricated by a centrifugation method. Biomaterials.

[28] Lu X., Wang C., Wei Y. (2009). One-dimensional composite nanomaterials: Synthesis by electrospinning and their applications. Small.

[29] Venugopal J.R., Low S., Choon A.T., Kumar A.B., Ramakrishna S. (2008). Nanobioengineered electrospun composite nanofibers and osteoblasts for bone regeneration. Artif. Organs.

[30] Lim J.M., Moon J.H., Yi G.R., Heo C.J., Yang S.M. (2006). Fabrication of one-dimensional colloidal assemblies from electrospun nanofibers. Langmuir.

[31] Hoppe A., Güldal N.S., Boccaccini A.R. (2011). A review of the biological response to ionic dissolution products from bioactive glasses and glass-ceramics. Biomaterials.

[32] Pham Q.P., Sharma U., Mikos A.G. (2006). Electrospun Poly(ε-caprolactone) Microfiber and Multilayer Nanofiber/Microfiber Scaffolds: Characterization of Scaffolds and Measurement of Cellular Infiltration. Biomacromolecules.

[33] Roosa S.M.M., Kemppainen J.M., Moffitt E.N., Krebsbach P.H., Hollister S.J. (2010). The pore size of polycaprolactone scaffolds has limited influence on bone regeneration in an *in vivo* model. J. Biomed. Mater. Res. Part A.

[34] Liverani L., Boccaccini A.R. Electrospinning with benign solvents: Feasibility study and versatile use of poly(epsilon-caprolactone) fibers. Proceedings of 10th World Biomaterials Congress.

[35] Wutticharoenmongkol P., Sanchavanakit N., Pavasant P., Supaphol P. (2006). Preparation and characterization of novel bone scaffolds based on electrospun polycaprolactone fibers filled with nanoparticles. Macromol. Biosci..

[36] Gönen S.Ö., Taygun M.E., Küçükbayrak S. (2016). Fabrication of Bioactive Glass Containing Nanocomposite Fiber Mats For Bone Tissue Engineering Applications. Compos. Struct..

[37] Kouhi M., Morshed M., Varshosaz J., Fathi M.H. (2013). Poly(epsilon-caprolactone) incorporated bioactive glass nanoparticles and simvastatin nanocomposite nanofibers: Preparation, characterization and *in vitro* drug release for bone regeneration applications. Chem. Eng. J..

[38] Catledge S.A., Clem W.C., Shrikishen N., Chowdhury S., Stanishevsky A.V., Koopman M., Vohra Y.K. (2007). An electrospun triphasic nanofibrous scaffold for bone tissue engineering. Biomed. Mater..

[39] Ghasemi-Mobarakeh L., Prabhakaran M.P., Morshed M., Nasr-Esfahani M.-H., Ramakrishna S. (2008). Electrospun poly(ε-caprolactone)/gelatin nanofibrous scaffolds for nerve tissue engineering. Biomaterials.

[40] Gaharwar A.K., Nikkhah M., Sant S., Khademhosseini A. (2014). Anisotropic poly(glycerol sebacate)-poly(ε-caprolactone) electrospun fibers promote endothelial cell guidance. Biofabrication.

[41] Kokubo T., Takadama H. (2006). How useful is SBF in predicting *in vivo* bone bioactivity?. Biomaterials.

[42] Aguiar H., Serra J., González P., León B. (2009). Structural study of sol–gel silicate glasses by IR and Raman spectroscopies. J. Non. Cryst. Solids.

[43] Zheng K., Solodovnyk A., Li W., Goudouri O.-M., Stähli C., Nazhat S.N., Boccaccini A.R. (2015). Aging Time and Temperature Effects on the Structure and Bioactivity of Gel-Derived 45S5 Glass-Ceramics. J. Am. Ceram. Soc..

[44] Lin H.M., Lin Y.H., Hsu F.Y. (2012). Preparation and characterization of mesoporous bioactive glass/polycaprolactone nanofibrous matrix for bone tissues engineering. J. Mater. Sci. Mater. Med..

[45] Jo J.H., Lee E.J., Shin D.S., Kim H.E., Kim H.W., Koh Y.H., Jang J.H. (2009). *In vitro*/*in vivo* biocompatibility and mechanical properties of bioactive glass nanofiber and poly(ε-caprolactone) composite materials. J. Biomed. Mater. Res. Part B.

